# Hypermethylation of DLG3 Promoter Upregulates RAC1 and Activates the PI3K/AKT Signaling Pathway to Promote Breast Cancer Progression

**DOI:** 10.1155/2021/8428130

**Published:** 2021-11-02

**Authors:** Bingbing Liu, Yanning Xu, Lin Zhang, Xue Yang, Ling Chen, Yixin Liu

**Affiliations:** Department of Pathology, Tianjin Central Hospital of Gynecology Obstetrics (Tianjin Key Laboratory of Human Development and Reproductive Regulation), Tianjin 300100, China

## Abstract

**Objective:**

This investigation aimed to figure out the relation between discs large homolog 3 (DLG3) expression and the progression and prognosis of breast cancer (BC).

**Methods:**

qRT-PCR was utilized for confirming DLG3 expression and RAC1 mRNA expression in BC tissues and cells. Subsequently, after overexpression or interference of DLG3, the changes of the biological activities of BC cells, including cell proliferation, migration, invasion, and apoptosis, were detected through CCK-8, colony formation assay, wound healing assay, transwell assay, and flow cytometry, respectively. Furthermore, western blotting was utilized to measure the protein expression of DLG3 and RAC1, as well as related proteins of epithelial-mesenchymal transition (EMT) and the PI3K/AKT signaling pathway.

**Results:**

At both cellular and tissue level in BC, DLG3 was downregulated and methylation level was upregulated; RAC1 showed an opposite change and was of a negative correlation with DLG3. In MCF-7 and HCC1937, we found that the upregulation of DLG3 could inhibit RAC1 expression as well as cell proliferation, invasion, migration, and EMT, while promoting apoptosis. Also, DLG3 inhibited the activation of the P13K/AKT pathway.

**Conclusion:**

Hypermethylation of DLG3 promoter upregulates RAC1 and activates the PI3K/AKT pathway, thus promoting BC progression. This conclusion provides ideas and experimental basis for improving and treating BC patients.

## 1. Introduction

Among all malignant tumors in females, breast cancer (BC) is described as the most common one [1], and it is the second most fatal cancer accounting for 14% of all cancer-related deaths [2]. The incidence of BC, as in most other countries, is high in the Chinese female population, with new cases accounting for 12.2% of global new cases; Chinese BC patients account for 9.6% of all BC-caused deaths in the world [3]. BC is usually triggered by a combination of environmental, physical, and biological factors. Biological factors refer to heredity, infection, or gene mutation, which probably lead to the transformation of a normal breast cell into a cancer cell [4]. BC, a highly heterogeneous disease, has been clinically divided into three subtypes according to the expression of estrogen receptor (ER), progesterone receptor (PR), and human epidermal growth factor receptor (HER2), namely, luminal BC (ER+/PR+ and HER2−) and HER2-positive BC (HER2+), as well as triple negative BC (ER−, PR−, and HER2−) [5]. Treatment options for BC depend on the specific molecular subtype. However, while surgical techniques and treatment regimens have made advancement, BC patients are still prone to recurrence and metastasis, which are the main cause of their death [2, 6]. Therefore, it is vital to deeply understand the molecular mechanism of BC progression, so as to realize the prevention, diagnosis, and treatment of this disease.

Increasing studies have discovered that epigenetic instability affects the occurrence and development of malignant tumors [7]. DNA methylation is an epigenetic modification which has been studied the earliest and most intensively, and abnormal DNA methylation is also one of the earliest discovered indicators related to tumor cell proliferation, migration, and invasion [8, 9]. Many laboratory and clinical data have confirmed that abnormal activity of tumor cells induces abnormal hypermethylation of the whole genome, thus aggravating tumor progression [10]. In mammalian cells, DNA methylation occurs on the 5-carbon position of cytosine in CpG dinucleotides, and its change is related to many important gene events as well as malignant tumors' occurrence and development [11]. The increase of gene promoter methylation is considered to be a marker of gene expression inhibition. Discs large homolog 3 (DLG3), also known as SAP102, is a member of the membrane-associated guanylate kinase family (MAGUKs) [12]. Directed trafficking of DLG3 plays a crucial role in different types of polarized cells and in the establishment and maintenance of apical cell junctions. In recent studies, by comparison with the normal tissues, BC and neuroblastoma tissues showed higher methylation level of DLG3 [13, 14]. Collectively, DLG3 may be associated with BC development, but its biological function and specific molecular mechanism in BC remain unclear and, therefore, need to be further investigated.

RAC1 is a member of the Rho GTPase family, which encodes a GTPase belonging to the Ras superfamily of small GTP-binding proteins. Members of this superfamily can regulate a variety of cell activities including cell growth, cytoskeleton remodeling, protein kinase activation, and tumor angiogenesis [15], and Ras-related GTPase in the Rho family is closely related to cytoskeleton remodeling [16, 17]. RAC1 significantly affect cell motility, invasion, and metastasis and is of a close relation with the promotion of the epithelial-mesenchymal transition (EMT) of tumor cells [18–20]. It has been reported that the increase of RAC1 expression promotes the occurrence and progress of BC [21], but whether DLG3 can regulate RAC1 expression in BC remains unclear.

This study was designed to explore the potential role of DLG3 in BC progression; our results showed that DLG3 hypermethylation could upregulate RAC1 expression and activate the PI3K/AKT signaling pathway and promote the malignant development of BC cells. This study contributes to the understanding of the mechanism of BC development and to an advance of effectiveness of the treatment for BC.

## 2. Materials and Methods

### 2.1. Collection and Treatment of Clinical Specimens

BC and paracancerous (normal) tissues of patients undergoing radical mastectomy in our hospital from January 2019 to December 2019 were collected. All patients, with BC as the primary lesion confirmed by pathological examination, had no chemotherapy and radiotherapy before their surgery and had no history of major systemic diseases. Their informed consent and an approval from the Medical Ethics Committee of Tianjin Central Hospital of Gynecology Obstetrics (2021KY004) were obtained.

### 2.2. Cell Culture

Human normal breast cells (MCF10A) and BC cells (MCF-7, MDA-MB-231, SK-BR-3, and HCC1937) were cultured after purchasing from the cell bank of Shanghai Institute of Biochemistry and Cell Biology, Chinese Academy of Sciences (Shanghai, China). The culture conditions were as follows: RPMI-1640 medium with a supplement of 10% fetal bovine serum, 100 U/ml penicillin, and 100 *μ*g/ml streptomycin, 37°C and 5% CO_2_. The cells were digested and passaged with 0.25% trypsin every 2 to 3 days. The cells in the logarithmic phase were taken for follow-up experiments.

### 2.3. Cell Transfection

On completion of the digestion of collected MCF-7 and HCC1937 cells in the log phase by 0.25% trypsin, the cells were seeded in 6-well plates (1 × 10^6^ cells/well). With the confluency of 80%–90%, they were transfected according to the Lipofectamine TM 2000 kit instructions. DLG3 interference fragment DLG3-siRNA and overexpression vector DLG3-pcDNA were designed and synthesized by Sangon Biotech (Shanghai, China). The cells were grouped into the NC group (without transfection), si-DLG3 group (with transfection of DLG3-siRNA), and oe-DLG3 group (with transfection of DLG3-pcDNA) and cultured for 48 hours.

### 2.4. Bisulfite Sequencing PCR

DNA in cells was obtained with a genomic DNA extraction kit, and bisulfite modification of DNA was performed on the basis of the DNA methylation kit. The TakaRaEpiTaqHS enzyme was used to amplify the modified DNA with the following cycling conditions: 10 s at 98°C, 30 s at 55°C, and 30 s at 72°C for a total of 40 cycles. After purification and subcloning of the abovementioned PCR products into the pGEMTEasy vector and through blue-white screening, positive clones were sent for sequencing. QUMA and BIQ analyzer were introduced in the analysis of the methylation status of every clone. Primers used to amplify the DLG3 promoter fragment in BC tissues were upstream 5′-GTTTTTTAAATTTATTAATGGGATTTAGG-3′; downstream 5′-TCCCTCCCCAACCCAAAAAA-3′. Primers used in nested PCR for amplifying the promoter fragment on the luciferase reporter plasmid pGL3-DLG3 were lateral upstream 5′-GTTTTTTTTAAGGATTTAGG-3′; lateral downstream 5′-GTTTTAAATTGGGATTTAGG-3′; medial upstream 5′-GTTTTTTTTAAATTTAGG-3′; and medial downstream 5′-GTTTTTTTTAAATTGGGATTTAGG-3′.

### 2.5. CCK-8 Method

We seeded and cultured the cells in 96-well plates (density: 1 × 10^4^ cells/well) with the addition of CCK-8 solution (10 *μ*l/well) for 0, 24, 48, and 72 hours. Subsequently, on completion of further 2-hour culture in an incubator, the cells were collected. The absorbance at 450 nm was detected by using an automatic enzyme-labeled instrument. We set 3 repetitions for each culture time, and the experiment was repeated 3 times.

### 2.6. Cell Colony Formation Experiment

On completion of digestion by trypsin and subsequent preparation of a single-cell suspension, BC cell concentration was determined and then adjusted to 1000 cells/ml. Then, the suspension was inoculated evenly and cultured aseptically in 6-well plates. The media were changed every 3 days, and the culture was terminated when visible clones appeared. After washed by PBS twice, the fixation step of the cells by 4% paraformaldehyde and subsequent 30-min staining by GIMSA were carried out. The final step was to calculate the colony formation rate.

### 2.7. Flow Cytometry Detection

On completion of the rinsing step utilizing PBS, centrifugation (1000r/min, 2 min) for the cells was followed to adjust cell concentration to 1.5 × 10^5^ cells/mL. Subsequently, resuspension of the cells was prepared with 195 *μ*l Annexin V-FITC binding solution, and then, after 5 *μ*L Annexin V-FITC was added and mixed, 10-min culture was carried out at ambient temperature in the dark. After that, this mixture was added with 10 *μ*l PI staining solution and gently mixed, followed by placing it in the dark for 10 min at ambient temperature. Then, the cells were resuspended again with 200 *μ*l Annexin V-FITC binding solution. The final step was to analyze the stained samples by using a flow cytometer.

### 2.8. Transwell Experiment

The transwell upper chamber coated with Matrigel was placed in an incubator with the following conditions: 37°C, 5% CO_2_, for about 30 min. Then, a 24-hour culture was performed with an addition of 100 *μ*l transfected cell suspension in the upper chamber and 500 *μ*l DMEM supplemented with 5% fetal bovine serum in the lower chamber. After that, the inserts were taken out, followed by fixation with 4% paraformaldehyde, staining with 0.1% crystal violet, and rinsing with PBS. The final step was to wipe off the noninvaded cells in the upper chamber with a cotton swab. An orthostatic microscope was utilized for photographing and Image J 1.8.0 for data analysis.

### 2.9. Wound Healing Assay

After transfection, another 12-hour culture of the cells was carried out; after the cells were stable, the wound healing assay was performed in 6-well plates. The sterilized tip of the transfer tube was used to draw a line with uniform width at the maximum diameter of each well. On completion of the removal of the scattered from the scratches by gently washing with PBS buffer, further culture was carried out and completed in a constant-temperature incubator. The inverted microscope was used for observation and photographing on the day (0 h) and 48 h after the drawing. The results were quantitatively analyzed by Adobe Illustrator software.

### 2.10. qRT-PCR

Following the isolation of total RNA from BC cells and tissues utilizing Trizol reagent (Invitrogen) in accordance with the manufacturer's steps, the cDNA transcription kit (ABI) was applied for reverse transcription that converted RNA to cDNA. With the application of the SYBRH Select Master Mix (Invitrogen), parameters for qRT-PCR were 95°C for 2 min and then 40 cycles of 95°C, 15 s, 60°C, 1 min, and 72°C, 30 s. With GAPDH for normalization, quantitative analysis utilizing the 2^−ΔΔCt^ method was conducted. The primers used were.

DLG3,5′-GCTTCGGCAGCATACTAAAAT-3′ and 5′-CGCTTCACGAATTTGCGTGTCAT-3′; RAC1, 5′-CTTGACATGATTAGCTGGCATGATT-3′ and 5′-CCTGTGCAATGCCGTGTAGA-3′; and GAPDH, 5′-AACGGATTTGGTCGTATTG-3′ and 5′-GGAAGATGGTGATGGGATT-3′.

### 2.11. Western Blot Experiment

After proteins were extracted from the cells by utilizing RIPA buffer, BCA was applied for protein quantification. SDS-PAGE was followed by protein transfer to PVDF membranes, and then, the 2-hour blocking step utilizing 5% skimmed milk was conducted. After that, at 4°C, the membranes were incubated with primary rabbit polyclonal antibody DLG3 (ab152132, 1 : 1000), rabbit polyclonal antibody RAC1 (ab155938, 1 : 1000), mouse monoclonal antibody E-cadherin (ab76055, 1 : 1000), mouse monoclonal antibody vimentin (ab8978, 1 : 1000), rabbit monoclonal antibody N-cadherin (ab76011, 1 : 1000), mouse monoclonal antibody PI3K (ab140307, 1 : 1000), rabbit monoclonal antibody p-PI3K (ab245781, 1 : 1000), rabbit polyclonal antibody AKT (ab8805, 1 : 1000), rabbit polyclonal antibody p-AKT (ab38449, 1 : 1000), and rabbit monoclonal antibody GAPDH (ab181602, 1 : 1000). Secondary antibodies labeled with horse radish peroxidase (HRP) were then added to the membranes for another 2-hour incubation. The results were analyzed by using the chemiluminescence and gel imaging system. Then, the image was quantitatively determined by Image J (NIH).

### 2.12. Statistical Analysis

By utilizing SPSS 22.0, the results were statistically analyzed. Measurement data were expressed in the form of mean ± standard deviation (SD). Comparison between two groups was completed by the *t*-test, while comparison among three groups was carried out by one-way ANOVA. Every experiment was repeated three times or more. A statistically significant difference could be suggested if *P* < 0.05.

## 3. Results

### 3.1. Downregulation of DLG3 and Hypermethylation of Its Promoter Region in BC

The results of qRT-PCR and western blot confirmed that DLG3 mRNA and protein had lower expression in BC tissues (Figure 1(a) and 1(b)); at the cellular level, qRT-PCR also revealed the downregulation of DLG3 in BC cells in comparison with MCF10A (Figure 1(c)). Furthermore, bisulfite sequencing PCR indicated that by comparison with the normal group, the DNA methylation level of DLG3 in the BC tissue group showed a marked upregulation (Figure 1(d)); a similar increase was also found in BC cells (Figure 1(e)). The lowest DLG3 expression was found in MCF-7 and the highest in HCC1937. Therefore, these two kinds of BC cells were selected for the following experiments.

### 3.2. Overexpression of DLG3 Inhibits Proliferation and Promotes the Apoptosis of BC Cells

We confirmed the biological function of DLG3 in BC cells through gain- and loss-of-function assays. On completion of overexpression or knockdown of DLG3 in MCF-7 and HCC1937 cells, transfection efficiency was validated by qRT-PCR results (Figure 2(a)). In comparison with the NC group, the si-DLG3 group induced a significant promotion of proliferation and viability and an inhibition of apoptosis, while oe-DLG3 caused the opposite results (Figures 2(b)–2(d)). Taken together, the overexpression of DLG3 inhibited proliferation but promoted the apoptosis of BC cells.

### 3.3. Upregulation of DLG3 Inhibits Invasion, Migration, and EMT of BC Cells

Transwell, wound healing, and western blot assays were utilized for further investigating the biological function of DLG3 in BC cells. In comparison with the NC group, the si-DLG3 group showed a significant upregulation of invasion and migration; additionally, E-cadherin expression was decreased while vimentin and N-cadherin expression was increased after the knockdown of DLG3. The oe-DLG3 group had opposite changes (Figures 3(a)–3(e)). Taken together, the overexpression of DLG3 inhibited invasion, migration, and EMT of BC cells.

### 3.4. Upregulation of DLG3 Decreases RAC1 Expression

The results of qRT-PCR and western blot confirmed that RAC1 mRNA and protein had higher expression in BC tissues (Figures 4(a) and 4(b)); at cellular level, qRT-PCR also revealed the downregulation of RAC1 mRNA in BC cells in comparison with MCF10A (Figure 4(c)).

Subsequently, we explored the effect of DLG3 expression level on RAC1. The results of qRT-PCR indicated that, in comparison with the NC group, the si-DLG3 group showed a significant upregulation of RAC1 mRNA and protein, while the oe-DLG3 group caused opposite changes (Figures 4(d) and 4(e)). In addition, we used DNA methylation inhibitor 5-aza-DC to treat MCF-7 and HCC1937 cells. In comparison with the NC group, the 5-aza-DC group showed a markedly lower DNA methylation level of DLG3 and induced an increase of DLG3 expression and a decrease of RAC1 expression (Figures 4(g) and 4(h)). These results confirmed that DLG3 could regulate RAC1 expression in BC cells.

### 3.5. Inhibition of the PI3K/AKT Pathway by DLG3

Activation of PI3K/AKT is known to be closely related to BC, but its relation with DLG3 remains unclear.

In this study, western blot results showed (Figure 5) a reduction of p-PI3K and p-AKT protein expression levels in the oe-DLG3 group in comparison with the NC group and no significant differences between the two groups in PI3K and AKT expression, suggesting decreased ratios of p-PI3K/PI3K and p-AKT/AKT. In comparison with the NC group, an addition of PI3K/AKT pathway activator 746Y-P (740Y-P group) led to significant increases of p-PI3K and p-AKT protein expression levels and no marked differences in PI3K and AKT expression between the two groups, suggesting increased ratios of p-PI3K/PI3K and p-AKT/AKT. From further comparison between the oe-DLG3 group and oe-DLG3+740Y-P group, marked upregulation of p-PI3K and p-AKT expression was detected in the latter and no significant difference in PI3K and AKT expression between the two groups, indicating increased ratios of p-PI3K/PI3K and p-AKT/AKT. Taken together, these results confirmed that the inhibition of proliferation and metastasis of BC cells by DLG3 was achieved by suppressing PI3K/AKT pathway activation.

## 4. Discussion

Novel tools for diagnosing and predicting prognosis are required to treat more BC patients earlier and reduce the high mortality of BC. The biological effects of many cell polarity proteins in BC and other malignant tumors have been reported [22]. Previous studies have shown that DLG3 levels and its methylation showed an abnormal change in breast, renal, liver, lung, and ovarian cancers [23–25]. In this research, the downregulation of DLG3 and hypermethylation of its promoter region in BC were found. Recent studies have shown that the overexpression of DLG3 in glioblastoma can induce mitotic cell cycle arrest and apoptosis and leads to an inhibition of proliferation and migration but has no effect on invasion [13]. The inhibition of cells growth and adhesion by DLG3 has been reported to be achieved by regulating catenin. We confirmed that the overexpression of DLG3 inhibited BC cell proliferation, migration, and EMT, but promoted the apoptosis of cells.

Furthermore, we focused on the specific mechanism of the effects of DLG3 on the biological characteristics of BC cells. Many signaling pathways and genes have been mentioned as key points in cell activities, such as cell growth, proliferation, and gene expression regulation [26]. RAC1 belongs to the Rho GTPase family, and many studies have revealed that Rho GTPase pathways play a critical role in regulating tumor cell cytoskeleton reorganization and cell morphology and migration; a close relation of RAC1 with EMT of tumor cells is suggested [19, 27]. RAC1 also involves in regulating the migration of vascular endothelial cells and in regulating VEGF-mediated angiogenesis. The latter is achieved by the regulation of wild-type p53 expression by RAC1 [28]. Studies have reported that RAC1 expression is significantly upregulated in many tumors including ovarian [29], breast [30], and colorectal cancers [31]. In this research, we observed increased RAC1 expression levels in BC tissues and cells. In addition, there was a correlation between DLG3 and RAC1 expression. Specifically, in BC cells, the overexpression of DLG3 reduced the expression of RAC1 and treatment of 5-aza-DC also downregulated RAC1 expression. Collectively, RAC1 may act as a downstream target of DLG3 to mediate the role of DLG3 in BC.

The PI3K/AKT signaling pathway is a downstream signaling pathway of epidermal growth factor receptor, which is overexpressed in a variety of malignant tumors, such as breast [32], ovarian [33], lung [34], and liver cancers [35]. The activation rate of this pathway is at a high level in BC, and its abnormal activation can induce the proliferation and differentiation of tumor cells and can affect cell cycle [36, 37]. Additionally, the PI3K/AKT signaling pathway can promote tumor angiogenesis and, subsequently, invasion and migration of tumor cells, suggesting its participation in the biological behavior of various tumor cells [38, 39] and its impact on tumor progression. It has also been reported that this pathway not only induces the proliferation and differentiation of BC cells but also has a close relationship with BC invasion, migration, recurrence, and drug resistance [40]. In our study, the correlation between DLG3 and the PI3K/AKT signaling pathway was confirmed by western blot. Specifically, the overexpression of DLG3 could significantly reduce the ratios of p-PI3K/PI3K and p-AKT/AKT; the overexpression of DLG3 + PI3K/AKT activator 740Y-P could markedly upregulate the abovementioned ratios. Therefore, it is speculated that DLG3 can inhibit PI3K/AKT pathway activation.

## 5. Conclusions

To conclude, the hypermethylation of DLG3 and lowly expressed DLG3 are revealed in BC cells and tissues in vitro and in vivo; furthermore, the in-depth mechanism study confirms that the decrease of DLG3 expression level contributes to the upregulation of RAC1 and the abnormal activation of the PI3K/AKT pathway, thus affecting BC cell invasion, metastasis, and EMT. Our study still has some limitations, such as insufficient clinical samples and no subsequent animal experiments. Therefore, the reliability of this molecular mechanism is required to be further studied and confirmed. At present, there is a lot of related literature regarding epigenetics in BC in vivo. This study can deepen the understanding of the complex biological behaviors of BC cells and specific molecular mechanisms regulating BC cells, thus providing an experimental basis and strategies for the clinical treatment to improve the survival rate of BC patients.

## Figures and Tables

**Figure 1:** Downregulation of DLG3 and hypermethylation of its promoter region in breast cancer. (a) Measurement of DLG3 expression in breast cancer (BC) and paracancerous (normal) tissues by qRT-PCR; (b) evaluation of DLG3 protein expression in BC and normal tissues by western blot; (c) determination of DLG3 expression in BC cells and MCF10A by qRT-PCR; (d) bisulfite sequencing PCR results of methylation levels of DLG3 in BC and normal tissues; and (e) bisulfite sequencing PCR results of methylation levels of DLG3 in BC cells and MCF 10A. ^*∗*^*P* < 0.05; ^∗∗^*P* < 0.01.

**Figure 2:** High expression of DLG3 inhibits proliferation and promotes the apoptosis of breast cancer cells. (a) Measurement of DLG3 expression in breast cancer cells transfected with DLG3-siRNA and overexpression vector by qRT-PCR; (b) evaluation of proliferation by CCK-8; (c) determination of colony formation; and (d) assessment of apoptosis by flow cytometry. ^∗∗^*P* < 0.01 vs. NC group.

**Figure 3:** Upregulation of DLG3 inhibits EMT, migration, and invasion of breast cancer cells. (a-b) Transwell-based assessment of cell invasion; (c-d) wound healing assay-based evaluation of cell migration; (e) detection of EMT-related proteins in MCF-7 cells by western blot. ^∗∗^*P* < 0.01 vs. NC group.

**Figure 4:** DLG3 can inhibit RAC1 expression in breast cancer cells. (a) qRT-PCR-based assessment of RAC1 expression in paracancerous tissues (normal) and breast cancer (BC) tissues; (b) evaluation of RAC1 protein expression in BC and normal tissues by western blot; (c) determination of RAC1 expression in BC cells and MCF10A by qRT-PCR; (d) qRT-PCR-based measurement of RAC1 expression in BC cells after the overexpression or interference of DLG3; (e) western blot-based assessment of RAC1 protein expression in BC cells after the overexpression or interference of DLG3; after treatment of DNA methylation inhibitor 5-aza-dC, (f) DLG3 methylation level in the cells was measured by bisulfite sequencing PCR; (g) DLG3 and RAC1 expression was measured by qRT-PCR; and (h) western blot was utilized for detecting DLG3 and RAC1 protein expression in MCF cells. ^*∗*^*P* < 0.05; ^∗∗^*P* < 0.01.

**Figure 5:** Inhibition of the PI3K/AKT pathway by DLG3. Western blot-based assessment of p-PI3K, PI13K, AKT, and p-AKT in MCF-7 cells after the overexpression of DLG3 (oe-DLG3 group) or after the overexpression of DLG3 + and the oe-DLG3+PI3K/AKT activator 740Y-P (oe-DLG3+740-Y-P group).

## Data Availability

No datasets were generated or analyzed during the current study.
